RETRACTED

# MiR-502 Suppresses TNF-*α*-Induced Nucleus Pulposus Cell Apoptosis by Targeting TARF2

**DOI:** 10.1155/2021/5558369

**Published:** 2021-04-01

**Authors:** Zhao Guo, Wen-Shan Gao, Yun-Fei Wang, Fei Gao, Wei Wang, Wen-Yuan Ding

**Affiliations:** ^1^Orthopedics Department, The Third Hospital of Hebei Medical University, Shijiazhuang, Hebei 050051, China; ^2^Orthopedics Department, Affiliated Hospital of Hebei University, Baoding, Hebei 071002, China

## Abstract

Intervertebral disc degeneration (IVDD) is a common cause of low back pain. This study is aimed at investigating the role of microRNAs (miRNAs) in regulating human nucleus pulposus (NP) cell injury induced by tumor necrosis factor- (TNF-) *α* in IVDD. In this study, we induced NP cells with 20 ng/mL TNF-*α* in vitro, which promoted the obvious apoptosis of NP cells and the activation of nuclear transcription factor (NF)-*κ*B. In contrast, using the specific NF-*κ*B inhibitor BAY 11-7082 to treat cells greatly impaired the activation of NF-*κ*B and increased the sensitivity of NP cells to TNF-*α*-induced apoptosis. Moreover, both TNF-*α* and BAY 11-7082 treatments were associated with marked miRNA dysregulation, with miR-502 being upregulated by TNF-*α* treatment and downregulated by BAY 11-7082 treatment, respectively. And the overexpression of miR-502 enhanced NF-*κ*B activation and suppressed apoptosis of human NP cells induced by TNF-*α*, whereas the opposite was observed following miR-502 inhibition. Last, through bioinformatic analyses and luciferase reporter gene experiments, we identified TRAF2, an important activator of NF-*κ*B, as a miR-502 target gene. Similarly, siRNA-mediated knockdown of the TRAF2 expression also suppressed TNF-*α*-induced apoptosis and enhanced NF-*κ*B activation. Our findings provide evidence indicating that miR-502 is a key regulator of apoptosis of human NP cells induced by TNF-*α* by targeting TRAF2 and activating NF-*κ*B.

## 1. Introduction

Intervertebral disc degeneration (IVDD) is a serious form of degenerative spinal disease that markedly lowers the quality of life of affected individuals and significantly aggravates social and economic burdens [1, 2]. Unfortunately, the etiology of IVDD remains unclear. Reductions in the functionality and number of nucleus pulposus (NP) cells are known to be associated with IVDD incidences [3, 4], and excessive TNF-*α*-induced apoptosis of NP cells is considered to be a vital driver of this disease [3]. Cell apoptosis is a complex and tightly regulated process that can be induced through intracellular or extracellular signaling pathways (mitochondrial and death receptor pathways, respectively) [4]. By suppressing NP cell apoptosis, it may be possible to disrupt the development of the inflammatory lesions associated with IVDD. As such, identifying novel mechanisms to suppress apoptotic NP cell death represents a viable approach to prevent TNF-*α*-induced NP cell injury and relieving IVDD progression.

RETRACTED

IVDD is associated with elevated TNF-*α* level in affected patients [5]. As an inflammatory cytokine, TNF-*α* can induce apoptosis and inhibit the differentiation of NP cells in a context-dependent fashion [6], with robust evidence having confirmed the ability of TNF-*α* to directly drive the apoptotic death of NP cells and cells of the fibrous ring of the IVDD [7]. Following binding to cell surface receptors, TNF-*α* activates the transcription factor nuclear factor-*κ*B (NF-*κ*B), a main regulator of inflammatory, stress stimulation, oncogenic, and apoptotic signaling within cells [8]. NF-*κ*B activation in response to TNF-*α* or other compounds can often suppress cell apoptosis [9]; although in some cases, it can instead accelerate such apoptotic processes [10], highlighting the context-dependent nature of these signaling mechanisms. The precise role of TNF-*α*-induced NF-*κ*B activation in the context of human NP cell apoptosis, however, has yet to be elucidated.

MicroRNAs (miRNAs) are conserved RNAs that lack coding potential [11], yet are able to regulate cellular functionality in physiological and pathological contexts via controlling the specific target gene expression [12]. Binding to the 3′-untranslated region (3′-UTR) of a specific target gene and recruiting RNA-induced silencing complex (RISC), miRNAs can not only inhibit the translation of target mRNA but also promote mRNA degradation [13]. Individual miRNAs can often target hundreds or thousands of genes, giving them broad potential to regulate the survival, growth, and development of cells. Many miRNAs have been found to control TNF-*α*-induced NF-*κ*B activation, including miR-146, miR-199a, and miR-517a [14]. However, further research is warranted to fully define the list of potential miRNAs regulating cell apoptosis through this signaling pathway.

This study explored the role of miRNA and the molecular mechanism of miRNA regulating NF-*κ*B activation affecting TNF-*α*-induced apoptosis of human NP cells. Furthermore, the upstream regulatory mechanism of NF-*κ*B activation was studied by using the specific NF-*κ*B inhibitor BAY 11-7082 [15] treatment, the specific small interfering RNA transfection, and miRNA microarray assay in context of TNF-*α* treatment inducing the apoptosis of human NP cells. The ultimate goal was to elucidate the molecular mechanisms by which miRNA-502 inhibits the TRAF2 expression and thereby modulates NF-*κ*B signaling and the apoptosis of human NP cells response to TNF-*α* signaling.

RETRACTED

## 2. Materials and Methods

### 2.1. Cell Cultures

Human NP tissues obtained from patients undergoing discectomy from the Third Hospital of Hebei Medical University. NP cells were isolated from the NP tissues as described previously [16]. Culture human NP cells in 6-well plates in Dulbecco's Modified Eagle's Medium (DMEM; Gibco, NY, USA) contain 10% fetal bovine serum (FBS; Gibco) in a 37°C humidified 5% CO_2_ incubator. Seeded cells were either treated directly with TNF-*α* (20 ng/mL, Sigma–Aldrich) for 6 h or were first pretreated for 1 h with BAY 11-7082 (60 *μ*M, Beyotime, Nantong, China) prior to the addition of 20 ng/mL TNF-*α* for 6 h. Untreated cells served as controls, and experiments were conducted on triplicate samples. All of the experiments protocols were approved by the Ethics Committee of Third Hospital of Hebei Medical University.

### 2.2. Apoptosis Assay

TUNEL staining, flow cytometry, and caspase 3/7 activation assays were used to measure cellular apoptosis. For TUNEL staining, the DeadEnd™ Fluorometric TUNEL System (Promega, CA, USA) was used on the basis of the manufacturer's instructions. The Caspase-Glo® 3/7 Assay Kit (Promega) was used to assess caspase 3/7 activation. Human NP cell apoptosis was evaluated by flow cytometric analysis (Gallios, Beckman Coulter) of TUNEL/DAPI dual-staining (Invitrogen, CA, USA) based on the manufacturer's instructions.

### 2.3. miRNA Microarray Assay

Evaluation of differentially expressed miRNAs in treated cells uses commercial miRNA microarrays which contain 1900 miRNA-specific probes in the Sanger miRBase database (v21.0). All microarray hybridization studies were conducted by LC Sciences Biotech Company (Hangzhou, China). Hybridized chips were then washed and analyzed with an Axon 4000B laser scanner (Axon Instruments), with chips being scanned at a 10 *μ*m pixel size with Cy3 gain set to 460 nm and Cy5 gain set to 470 nm. Extract and analyze data from these analyses using ArrayPro ™ software with morphological filters (Media Cybernetics).

### 2.4. Cell Transfection

Human NP cells were transfected with miR-502 mimics, inhibitors, or appropriate control oligomers (Biomics Biotech, Nantong, China) for 24 h (100 nmol/L) prior to TNF-*α* treatment.

### 2.5. NF-*κ*B Activation Assay

A pGL4.32 [luc2P/NF-*κ*B-RE/Hygro] vector containing five NF-*κ*B response element (NF-*κ*B-RE) copies driving luciferase reporter gene (luc2P) expression was purchased from Promega (USA). Cells were cultured in 24-well plates until 70% fusion was achieved. Cells were then transfected with 0.5 *μ*g pGL4.32 [luc2P/NF-*κ*BRE/Hygro] plasmid DNA with Lipofectamine 2000. Cells were then hatched 37°C overnight before treatment with or without TNF-*α* (20 ng/mL) for 6 h. A luciferase activity was then tested with a dual-luciferase reporter assay system (Promega) on the basis of the manufacturer's instructions, with Renilla luciferase activity being used for normalization purposes and with all data being reported compared to the medium control.

RETRACTED

### 2.6. Analysis of p65 Phosphorylation

NF-*κ*B p65/RelA protein phosphorylation was assessed to gauge intracellular NF-*κ*B activation with the NF-*κ*B/p65 Phospho Tracer Immunoassay Kit (Abcam, Cambridge, UK) based on the manufacturer's instructions. In brief, after stimulation, cells were washed using PBS and were probed overnight at 4°C with an initial antibody. Subsequently, the cells were incubated with a corresponding secondary antibody. Substrate solution was then added for 30 minutes, and a plate reader (Biotek, VT, USA) was used to quantify cellular fluorescence.

### 2.7. Identification of miRNA Target Genes

Putative miRNA target genes were identified using the TargetScan (http://www.targetscan.org), Miranda (http://www.microrna.org/), and Pictar (http://pictar.mdc-berlin.de/) tools.

### 2.8. Luciferase Activity Assay

Wild type (WT) or mutated (MUT) versions of the TRAF2 3′-UTR sequence which contains the putative miR-502 binding site were cloned into the pGL3-control-mcs2 reporter vector by ligating them into EcoRI and PstI sites. Reporter assays were then conducted by plating 293 T cells in 24-well plates, transfecting them with the appropriate plasmids and miRNA constructs and harvesting them 48 h later for analysis using a dual-luciferase reporter assay system (Promega). Firefly luciferase activity was normalized.

### 2.9. qPCR

A Small RNA Reagent (TaKaRa Bio, Inc., Otsu, Japan) was used to extract miRNAs and other small RNAs from target cells based on the manufacturer's instructions, after which reverse transcription was conducted with a SYBR PrimeScript™ miRNA RT-PCR kit (Clontech, CA, USA). A SYBR Premix Ex Taq kit (TaKaRa) was then used to conduct qPCR on a Q6 system (ABI, NY). Use the 2^−*ΔΔ*Ct^ method to assess the relative gene expression.

### 2.10. Western Blotting Analysis

RIPA buffer (Beyotime, Nantong, China) was used to lyse cells, after which Western blot was conducted according to standard protocols using the following primary antibodies specific: GAPDH (Cat# 3683, Cell Signaling Technology, MA, USA), p-IKK (Cat# 2078), PARP (Cat# 5625), and TRAF2 (Cat# 2141). HRP-conjugated secondary antibodies were also purchased from Cell Signaling Technology, while anti-APAF1 (Cat# ab2001) was purchased from Abcam (Hercules, CA, USA).

RETRACTED

### 2.11. Statistical Analysis

All statistical analyses were performed using SPSS V19.0 (IBM, NY, USA), and the data were presented as mean ± standard deviation (SD). Data were compared using Student's tests or appropriate one-way analysis of variance, with *P* < 0.05 as the threshold of significance.

## 3. Results

### 3.1. NF-*κ*B Inhibition Enhances the Apoptosis of Human NP Cells

Human NP cells treated with TNF-*α* for 6 h moderately enhanced apoptosis (Figures 1(a) and 1(b)) and caspase 3/7 activity (Figure 1(c)). Furthermore, NF-*κ*B activation (Figure 1(d)) and NF-*κ*B p65 phosphorylation (Figure 1(e)) were enhanced by this treatment.

To investigate how NF-*κ*B influences TNF-*α*-induced apoptosis in human NP cells, we pretreated human NP cells with the NF-*κ*B-specific inhibitor BAY 11-7082. As demonstrated in Figures 1(d) and 1(e), BAY 11-7082 treatment significantly suppressed NF-*κ*B activation and p65 phosphorylation in these cells with TNF-*α* treatment. BAY 11-7082 treatment also markedly decreased the phosphorylation of inhibitor of NF-*κ*B kinase (IKK), an upstream regulator of this pathway. Correspondingly, cell apoptosis was also markedly increased in BAY 11-7082-treated NP cells following TNF-*α* treatment (Figures 1(a)–1(c)).

### 3.2. miRNA-502 Was Significantly Increased in TNF-*α*-Stimulated Human NP Cells

In an effort to determine which miRNAs serve as regulators of human NP cell apoptosis and NF-*κ*B signaling in response to TNF-*α* treatment, we assessed differential miRNA expression patterns in these cells using commercial miRNA microarrays. We identified 27 significantly differentially expressed miRNAs in the IVDD tissues compared with the normal tissues (*n* = 5). In these miRNAs, 13 were upregulated, and 14 were downregulated (Figure 2(a)). Similarly, compared with untreated human NP cells, we identified 27 miRNAs that were differentially expressed in TNF-*α*-stimulated NP cells (*n* = 3 for each group) (Figure 2(b)). Furthermore, qPCR results further demonstrated that miRNA-502 was significantly higher in IVDD tissues and TNF-*α*-stimulated human NP cells (Figure 2(d)) than their corresponding to normal tissues (*P* < 0.01, Figure 2(c)) and control (*P* < 0.001, Figure 2(c)), respectively.

### 3.3. MiR-502 Regulates TNF-*α*-Induced NF-*κ*B Activation and Apoptosis in Human NP Cells

NF-*κ*B signaling is known to influence the expression of miR-502 [17], whether miR-502 can inversely impact NF-*κ*B signaling through feedback mechanisms that remain to be established. Accordingly, we next transfected human NP cells with a miR-502 mimic prior to TNF-*α* stimulation, which resulted in a 22.5-fold rise in the expression of this miRNA relative to control cells (Figure 3(a)). The overexpression of miR-502 significantly enhanced NF-*κ*B activation (Figures 3(b) and 3(c)) and suppressed the TNF-*α*-induced apoptosis, as evidenced by reduced apoptotic cell numbers (Figures 3(d) and 3(e)), decreased caspase 3/7 activation (Figure 3(f)), and levels of the proapoptotic proteins, apoptotic protease activating factor-1 (APAF1), and cleaved poly ADP-ribose polymerase (PARP). In contrast, knockdown of the miR-502 expression by inhibitor negatively affected NF-*κ*B activation and enhanced TNF-*α*-induced apoptosis (Figure 3(g)). These findings suggested that miR-502 was positively correlated with NF-*κ*B.

RETRACTED

### 3.4. TRAF2 Is an miR-502 Target Gene in Human NP Cells

We next sought to identify miR-502 target genes likely to be associated with NF-*κ*B signaling by using online predictive tools. TRAF-associated NF-*κ*B activator (TRAF2, also taken for TRAF-Interacting protein) was identified as one such putative target gene (Figure 4(a)). In accordance with this prediction, the miR-502 overexpression was linked to the reduced TRAF2 expression at the mRNA level (*P* > 0.05, Figure 4(b)), as well as significant decreases in the TRAF2 expression at the protein level (Figure 4(c)). A luciferase reporter assay further confirmed that miR-502 mimic transfection was sufficient to suppress WT TRAF2 3′-UTR reporter activity by 65%, whereas no such suppression was observed for a mutated TRAF2 3′-UTR promoter. These results suggest that miR-502 is capable of binding to this predicted site within the TRAF2 3′-UTR and thereby regulating the translation of this mRNA (Figure 4(d)). Furthermore, qPCR data revealed changes in miR-502 and TRAF2 expression in human NP cells following TNF-*α* treatment that were consistent with this regulatory relationship (Figure 4(e)).

### 3.5. TRAF2 Knockdown Enhances TNF-*α*-Induced NF-*κ*B Activation in Human NP Cells

TRAF2 has been shown to specifically suppress TNF-*α*/TNFR-mediated NF-*κ*B activation [18]. Thus, we hypothesized that miR-502 regulates the TRAF2 expression and thereby controls the activation of NF-*κ*B within NP cells. To confirm this hypothesis, we knocked down endogenous TRAF2 in human NP cells by transfection with a specific siRNA construct (Figure 5(a)). We confirmed that TRAF2 knockdown was associated with increased NF-*κ*B activation (Figure 5(b)) and suppression of TNF-*α*-induced cell apoptosis (Figures 5(c) and 5(d)). Together, these findings emphasized the important role of miR-502 as a regulator of apoptosis in NP cells based on its ability to target TRAF2 and thereby to modulate NF-*κ*B activation.

RETRACTED

## 4. Discussion

While TNF-*α* is a well-known inducer of apoptotic death in human NP cells, further research regarding the underlying molecular mechanisms governing this relationship is warranted. Accumulating evidence suggests that miRNAs are crucial regulators of cell survival, differentiation, and proliferation [19]; however, the specific roles of miRNAs in the context of human NP cell apoptosis remain to be fully characterized. Therefore, in the study, we investigated the functional role of miRNAs in the inflammatory environment, leading us to identify dozens of miRNAs that were differentially expressed in these cells following TNF-*α* treatment. Additional bioinformatic analyses confirmed these miRNAs to be associated with cellular apoptosis.

NF-*κ*B serves as a key regulator of apoptotic processes within cells, and NF-*κ*B activation modulates cell survival in a context-dependent fashion. In previous studies, RelA knockout has been linked to enhanced TNF-*α*-induced apoptosis in embryonic fibroblasts [19]. Similarly, the TNF-*α* stimulation of RelA^−/−^ mice has been shown to result in substantial hepatocyte apoptosis and eventual death [20]. NF-*κ*B influences the expression of key antiapoptotic factors including TRAF1, TRAF2, c-IAP1, c-IAP2, IEX-1 L, Bcl-xL, and Bfl-1/A1 [21]. In contrast to these findings, however, there is also evidence that NF-*κ*B activation can induce or accelerate cell apoptosis. For example, substantial NF-*κ*B activation is observed in apoptotic 293 T cells under serum starvation conditions. Furthermore, the observation that NF-*κ*B inhibition or inactivation is sufficient to abrogate p53-induced apoptosis indicates that p53-mediated NF-*κ*B activation promotes programmed cell death. BAY 11-7082 treatment has also been shown to suppress NF-*κ*B activation in a series of cell types. In this study, it is found that BAY 11-7082-mediated NF-*κ*B suppression decreased apoptotic death in human NP cells, suggesting that this may be a valuable treatment for patients with IVDD.

MiR-502 was upregulated in response to TNF-*α* treatment in NP cells, but downregulated in response to BAY 11-7082. NF-*κ*B has previously been shown to regulate the expression of miR-502, which is encoded on the X chromosome in mammals [22]. Abnormal miR-502 expression has been detected in a range of human cancers [23], and there is clear evidence that this miRNA regulates cell apoptosis in many contexts. In hepatocellular carcinoma, for example, miR-502 is among the most differentially regulated miRNAs in tumor cells, promoting apoptotic death of HCC cells by targeting apoptosis inhibitor 5. In contrast, we found that miR-502 suppressed apoptosis in human NP cells by targeting TRAF2 and thereby enhancing NF-*κ*B signaling activity. These findings thus indicate that miR-502 can modulate apoptotic signaling pathways in a range of contexts, resulting in diverse outcomes. For example, there is evidence that miR-502 targets caspase 3 and caspase 7 in lung cancer cells to prevent TNF-*α*-induced cell apoptosis [24], which is consistent with our findings. Indeed, we also observed increased caspase 3/7 activity in miR-502 knockdown cells, thus emphasizing the complex regulatory role of this miRNA in the context of apoptosis.

RETRACTED

TRAF2 has previously been shown to modulate NF-*κ*B activation in a context-dependent fashion in response to TNF-*α*/TRAF signaling. TRAF2 can interfere with the binding of other TRAF proteins, thereby disrupting NF-*κ*B activation in response to exogenous stimuli like TNF-*α* and LPS [24]. However, in other settings, TRAF2 promotes TRAF-mediated NF-*κ*B activation [25]. In addition, there is evidence that TRAF2 synergizes with TBK1 and IKK-*ε*, bringing them together with IKK complexes and thereby controlling NF-*κ*B activation. Therefore, we identified and validated TRAF2 as a miR-502 target gene, confirming that this miRNA modulates NF-*κ*B signaling, at least in part, by regulating the TRAF2 expression.

In conclusion, our findings emphasize the role of miR-502 as a regulator of apoptotic death of human NP cells in response to TNF-*α* stimulation based on its ability to target TRAF2 and thereby control NF-*κ*B activation.

## Figures and Tables

**Figure 1:** NF-*κ*B inhibition enhances the cell apoptosis of human NP cells. (a) Flow cytometric analysis (TUNEL/DAPI dual-staining) of apoptotic cell frequency. (b) Detection of TUNEL-positive cells by fluorescence microscopy (×10; DMi8, Leica, Germany). TUNEL-positive cells are shown in green, with DAPI staining (blue) showing cellular nuclei. (c) Caspase 3/7 activity. (d) NF-*κ*B activity. (e) Total and phosphorylated p65 levels. *n* = 5; different lower case letters indicate significant differences at *P* < 0.05.

**Figure 2:** The profiling of the differential miRNA expression in the IVDD patients compared with the control group and in TNF-*α*-treated and untreated NP cells. (a). A total of 27 miRNAs were differentially expressed in IVDD tissues and in normal tissues (*n* = 5 for each group). (b) A total of 27 miRNAs were differentially expressed in TNF-*α*-treated and untreated human NP cells for 6 h at 20 ng/mL (*n* = 3 for each group). Green: low expression; red: high expression. (c) The expression of miR-502 was detected in normal and IVDD tissues by qRCR. (d) The MiR-502 expression was measured in the NP cells with and without 20 ng/mL TNF-*α* by qRCR. ^∗∗^*P* < 0.01 and ^∗∗∗^*P* < 0.001.

RETRACTED

**Figure 3:** MiR-502 suppresses the TNF-*α*-induced apoptotic death of human NP cells. (a) Assessment of the miR-502 overexpression and knockdown efficiency. (b) Total and phosphorylated p65 levels in analyzed cells. (c) NF-*κ*B activity. (d) Flow cytometric analysis (TUNEL/DAPI dual-staining) of apoptotic cell frequency. (e) Detection of TUNEL-positive cells by fluorescence microscopy (×10; DMi8, Leica, Germany). TUNEL-positive cells are shown in green, with DAPI staining (blue) showing cellular nuclei. (f) Caspase 3/7 activity. (g) Western blot analysis of APAF1 and PARP levels at 48 h post-miR-502 mimic or inhibitor transfection, with GAPDH as a loading control. *n* = 5; different lower case letters indicate significant differences at *P* < 0.05.

**Figure 4:** TRAF2 is a target gene of miR-502. (a) A putative miR-502 binding site was identified in the TRAF2 3′-UTR. (b) The overexpression of miR-502 slightly decreased TRAF2 mRNA levels and (c) significantly decreased TRAF2 protein levels. (d) A luciferase reporter assay confirmed that miR-502 mimic transfection reduced the activity of a reporter containing the WT TRAF2 3′-UTR, whereas no such activity was observed when the putative miR-502 binding site within this reporter was mutated. (e) The expression of miR-502 and TRAF2 expression in human NP cells with TNF-*α* treatment. *n* = 5; different lower case letters indicate significant differences at *P* < 0.05.

**Figure 5:** TRAF2 silencing enhances NF-*κ*B activation and suppresses apoptotic death in human NP cells. (a) SiRNA-mediated TRAF2 knockdown. (b) NF-*κ*B activity. (c) Caspase 3/7 activity. (d) Flow cytometric analysis (TUNEL/DAPI staining) of apoptotic cell frequency. *n* = 5; different lower case letters indicate significant differences at *P* < 0.05.

## Data Availability

The datasets used and analyzed during the current study are available from the corresponding author on reasonable request.
